# Oxidative-Damaged Mitochondria Activate GABARAPL1-Induced NLRP3 Inflammasomes in an Autophagic-Exosome Manner after Acute Myocardial Ischemia

**DOI:** 10.1155/2022/7958542

**Published:** 2022-09-30

**Authors:** Tiechun Zhang, Dongyao Hou, Jianrong He, Xue Zeng, Ruixue Liu, Liangming Liu, Tao Li, Yingbin Xiao, Ruiyan Ma, He Huang, Chenyang Duan

**Affiliations:** ^1^Department of Anesthesiology, The Second Affiliated Hospital of Chongqing Medical University, Chongqing 400010, China; ^2^Department of Rehabilitation, the Fifth People's Hospital of Chongqing, Chinese Academy of Sciences, Chongqing 400062, China; ^3^Department of Shock and Transfusion, State Key Laboratory of Trauma, Burns and Combined Injury, Daping Hospital, Army Medical University, Chongqing 400042, China; ^4^Department of Cardiovascular Surgery, Xinqiao Hospital, Army Medical University, Chongqing 400037, China

## Abstract

**Objective:**

This study is aimed at identifying the potential diagnostic markers for circulating endothelial cells (CECs) for acute myocardial ischemia (AMI) and exploring the regulatory mechanisms of the selected biomarker in mitochondrial oxidative damage and vascular inflammation in AMI pathology.

**Methods:**

Utilizing the Gene Expression Omnibus dataset GSE66360, we scanned for differentially expressed genes (DEGs) in 49 AMI patients and 50 healthy subjects. To discover possible biomarkers, LASSO regression and support vector machine recursive feature elimination examinations were conducted. Using the GSE60993 and GSE123342 datasets and AMI rat models, the expression levels and diagnostic accuracy of the biomarkers in AMI were thoroughly verified. CIBERSORT was employed to evaluate the compositional patterns of 22 distinct immunological cell percentages in AMI according to combined cohorts. The oxidative-damaged mitochondria were detected by confocal microscopy observation of MitoTracker, ROS-DCFH-DA, and mCherry-GFP-LC3B.

**Results:**

In total, 122 genes were identified. The identified DEGs primarily contributed in arteriosclerosis, arteriosclerotic cardiovascular disorders, bacterial infectious disorder, coronary artery disease, and myocardial infarction. Nine features (NR4A2, GABARAPL1 (GEC1), CLEC4D, ITLN1, SNORD89, ZFP36, CH25H, CCR2, and EFEMP1) of the DEGs were shared by two algorithms, and GABARAPL1 (GEC1) was identified and verified as a diagnostic mitochondrial biomarker for AMI. Confocal results showed that there existed mitochondrial damage and oxidative stress in cardiac CMECs after AMI, and the blocked autophagy flux could be released by exosome burst in cardiac CMECs and blood CECs. Immune cell infiltration testing declared that elevated GEC1 expression in blood CECs was linked to the rise of monocytes and neutrophils. Functional tests revealed that high GEC1 expression in CMECs and CECs could activate the vascular inflammatory response by stimulating NLRP3 inflammasome production after AMI.

**Conclusion:**

Oxidative-damaged mitochondria in cardiac CMECs activate GEC1-mediated autophagosomes but block autophagy flux after AMI. The exfoliated cardiac CMECs evolve into abnormal blood CECs, and the undegraded GEC1 autophagosomes produce a large number of NLRP3 inflammasomes by exosome burst, stimulating the increase in monocytes and neutrophils and ultimately triggering vascular inflammation after AMI. Therefore, GEC1 in blood CECs is a highly specific diagnostic mitochondrial biomarker for AMI.

## 1. Introduction

Acute myocardial ischemia (AMI) is an inevitable process of most cardiovascular diseases. Presently, early risk assessment of acute myocardial ischemia, myocardial infarction, and the coronary syndrome is primarily based on initial history and physical examination findings and electrocardiogram and cardiac biomarker measurements [1, 2]. Myocardial ischemia involves neuroendocrine hormone activation, myocardial stretch, myocardial injury, cardiac matrix remodeling, inflammation, and other pathophysiological processes, each of which involves related biomarkers, such as cTnT, cTnI, CK-MB, H-FABP, and Hs-CRP [3]. However, the related biomarkers to reflect the mitochondrial damage after AMI have not been studied.

Although the present biomarkers for AMI have been in use, there exist different limitations to some extent. For example, the value of CK-MB is sensitive but has low specificity to AMI. The expressions of cTnT and cTnI usually do not increase until at least 6 h after the onset of symptoms, and their measurements have low sensitivity in the early phase of AMI. After myocardial necrosis, the value of cTnT remains elevated for 10-14 days, and it is hard to detect recurrent myocardial damage [4]. As mitochondria are very sensitive to ischemia and hypoxia injury, evaluation of mitochondrial damage and oxidative stress after AMI by appropriate biomarkers may timely and sensitively reflect the damage of ischemia and hypoxia to cardiac cells.

Approximately one-third of the size of adult cardiac cells is occupied by mitochondria [5]. Besides supplying the vast bulk of the energy consumed by the heart, the mitochondrial role encompasses diverse essential biological and regulating activities, including redox balance [6], biosynthesis, reactive oxygen species signaling, cell proliferation and apoptosis, ion homeostasis [7], protein quality control [8], and inflammatory processes [9]. The dysfunction of mitochondria is closely related to the severity of myocardial damage after acute myocardial ischemia (AMI) [10]. Unbalanced mitochondrial dynamics can activate oxidative stress, and an oxidative stress state can also induce mitochondrial dynamics imbalance and energy metabolism disorder. Therefore, preserving mitochondrial activity and targeting oxidative stress may be crucial for rescuing cardiac function following AMI [11]. However, the detection of mitochondrial cardiac injury in clinical AMI patients and the influence of mitochondrial injury on prognosis are not clear.

Recent studies have identified novel populaces of nonhematopoietic blood cells. Hardly observed in healthy blood, circulating endothelial cells (CECs), which are frequently characterized by the expression of membrane glycoprotein CD146, are elevated in a wide variety of clinical diseases, encompassing inflammatory, immunological, contagious, oncogenic, and cardiovascular disorders [12]. Increased CECs were found to anticipate worse cardiovascular outcomes in acute coronary syndromes; however, the underlying processes are still unexamined [13]. This work sought to uncover mitochondrial diagnostic markers in blood CECs that represent mitochondrial damage in cardiac tissue following AMI.

In the current study, we selected acute myocardial infarction as a typical clinical acute myocardial ischemic model to screen for mitochondrial-related genes with diagnostic efficacy in CECs of AMI using a machine learning algorithm and preliminary explore the regulatory mechanisms of the selected biomarkers to mitochondrial oxidative damage and vascular inflammation in AMI pathology.

## 2. Materials and Methods

### 2.1. Materials

Antibodies against GABARAPL1 (GEC1), CD146, LC3, GAPDH, TSG101, CD63, NLRP3, caspase-1, and interleukin- (IL-) 1*β* were acquired through Abcam (Cambridge, MA, USA). All PE- or FITC-conjugated secondary antibodies, MitoTracker Deep Red, Dynabeads, fetal bovine serum, and penicillin/streptomycin were obtained through Invitrogen (Carlsbad, CA, USA). Ad-mCherry-GFP-LC3 and ROS-DCFH-DA kit were acquired through Beyotime (Shanghai, China), while adenoviral vectors for GEC1 shRNA and AAV2-GEC1 shRNA were produced by GeneChem Technology (Shanghai, China). The endothelial basal medium EBM-2 medium kit was acquired through Lonza (Bern, Switzerland). Any other material was obtained through Sigma-Aldrich except if another source was mentioned.

### 2.2. Animal Model Preparation

Army Medical University, Research Institute of Surgery (Chongqing, China), supplied 220–270 g of male Sprague–Dawley rats. Left anterior descending (LAD) coronary artery occlusion was used to cause acute myocardial ischemia (AMI) in rats. The rats were sedated with 1% pentobarbital sodium (40 mg/kg, given i.p.) and oxygenated with a rodent ventilator (Shanghai Alcott Biotech Co., Ltd. China), a 6/0 suture, the LAD artery ligation. Effective blockage of the LAD was established by the existence of ST-segment elevation on the ECG (Guangzhou Sanrui Electronics Co., Ltd., China) and a coloration difference from bright red to light red in the ventricle. The musculature and skin were sutured separately for each layer, and the incisions were disinfected following assurance of effective shaping.

To reduce GEC1 expression in a rat model, adeno-associated virus- (AAV2-) shGEC1 was injected (5 × 10^13^ v.g/mL, 1 mL/kg) into rats via the tail vein two weeks before LAD.

### 2.3. Cell Culture and Hypoxia Treatment

CMECs were cultivated in an EBM-2 media kit enriched with 100 U/mL penicillin/streptomycin at 37°C in a humidified incubator under typical circumstances (5% CO2, 21% O2, and 74% N2). For hypoxic trials, CMECs were cultivated in serum-free Dulbecco's modified Eagle's media and then transmitted to a hypoxic culture compartment (MIC-101, Billups-Rothenberg, Del Mar, CA, USA) saturated with 94% N2, 5% CO2, and 1% O2 for 24 h.

### 2.4. Isolation of CECs, CMECs, and Monocytes

To isolate CECs and monocytes, 5 mL of blood from the abdominal aorta of rats including retrieved in a tube with ethylenediamine tetraacetic acid, diluted with 5 mL phosphate-buffered saline (PBS), and separated with rat peripheral blood lymphocyte isolation buffer (Solarbio, China) to retrieve mononuclear cell suspensions. Mononuclear cells were further separated by density gradient centrifugation to obtain monocytes or used to isolate CECs by magnetic-activated cell sorting (MACS). To isolate CECs by MACS, the mononuclear cell suspensions were first incubated with Dynabeads conjugated to anti-rat CD45 for 30 min at 4°C to deplete the cells and platelets expressing CD45. Next, the cell suspensions were incubated with Dynabeads conjugated to anti-rat CD146 for 30 min at 4°C for positive selection of CECs.

To isolate the CMECs, the hearts of rats were first minced, digested with 0.2% collagenase type II in Hank's basal salt solution for 45 min at 37°C with rotation, and filtered with a 70 *μ*m cell strainer to obtain single-cell suspensions. The CMECs were sorted positively from the suspension by MACS using Dynabeads conjugated to anti-rat CD146.

### 2.5. Screening of Differentially Expressed Genes (DEGs) and Diagnostic Value of Featured Biomarkers

The GSE66360, GSE60993, and GSE123342 datasets' matrix files were downloaded at http://www.ncbi.nlm.nih.gov/geo/. The GSE66360 dataset was utilized for DEG scanning, while the GSE60993 and GSE123343 databases were utilized to validate the expression patterns of the identified genes. The GSE66360 data were evaluated and represented using R/Bioconductor [14]. Individual gene expression was deemed to be altered when |log fold change| > 1.5; Welch's analysis of variance revealed a *p* value of 0.05 when comparing the mean normalized signal levels with the Bioconductor tool genefilter. To examine the role of DEGs, Bioconductor assessments of disease ontology (DO) enrichment, gene ontology (GO), and Kyoto Encyclopedia of genes and genomes (KEGG) were performed [15].

As described earlier [15], two distinct machine learning techniques, the least absolute shrinkage, and selection operator (LASSO) regression and the support vector machine recursive feature elimination (SVM-RFE) methods, were used to identify possible biomarkers among the DEGs. The overlapped genes between the two methods were chosen as possible predictive biomarkers, and their expression patterns were validated using the GSE60993 and GSE123343 databases.

Using mRNA expression information from the GEO public database, we developed a receiver operating characteristic (ROC) curve to evaluate the diagnostic accuracy of the chosen biomarkers. Furthermore, the area under the ROC curve (AUC) measure was utilized to estimate the diagnostic performance of distinguishing AMI samples from controls.

### 2.6. Discovery of Immune Cell Subtypes

As initially noted [15, 16], we used the bioinformatics tool (CIBERSORT) to calculate the relative ratios of immunological cell infiltration utilizing gene expression patterns in AMI to investigate immunity cell infiltration. Employing the “corrplot” R program, correlation analyses and visualization of 22 kinds of infiltrating immunological cells were done. Utilizing the “vioplot” tool in R, the variations in immunological cell infiltration between AMI and control samples were visualized using violin graphs.

### 2.7. Flow Cytometry Analysis

The cells were preserved and permeabilized for 20 min at 4°C utilizing fixation and permeabilization solution (BD Bioscience, Franklin Lakes, NJ, USA). Following two rinses with perm/wash buffer (BD Bioscience, Franklin Lakes, NJ, USA), the cell pellet was resuspended and blocked with 2% bovine serum albumin (BSA) at room temperature for 15 min, then incubated for 1 h at 4°C with the suggested quantity of antibody (CD146, GABARAPL1, or NLRP3). Before conducting the flow cytometric examination, the cells were treated with fluorochrome-conjugated secondary antibodies, then incubated for 30 min at 4°C in the dark and rinsed two times.

### 2.8. Immunofluorescence

Heart cell specimens were stained with immunofluorescence, as described previously [10]. The slides were preserved in 4% paraformaldehyde for 20 min, permeabilized with 0.1% triton-X 100 in PBS for 5 min, covered with 5% BSA/PBS for 1 h at 37°C, and then incubated for one night at 4°C with primary antibodies against GABARAPL1. The specimens were therefore rinsed with PBS containing 0.1% Tween-20 and incubated for 1 h at room temperature with FITC-conjugated mouse or rabbit secondary antibodies (Invitrogen, Carlsbad, CA, USA). After that, the specimens were rinsed prior to a final rinsing in 1X PBS and incubation with 4′,6-diamidino-2-phenylindole dye (BD Biosciences, Franklin Lakes, NJ, USA) (1 : 50) for 5 min at room setting. Using a confocal laser scanning microscope (Leica SP5, Germany), immunofluorescence was detected.

### 2.9. Western Blotting

The total protein was recovered by lysing the cells in ice-cold RIPA buffer, which was enriched using protease blockers (Beyotime, Shanghai, CHINA). The bicinchoninic acid (BCA) protein testing kit was utilized to get the results for protein contents (Beyotime, Shanghai, CHINA). After that, total protein was utilized for immunoblotting examinations utilizing the related antibodies, as was earlier [17]. The program Quantity One V 4.62 (Bio-Rad, Life Science, CA, USA) was utilized to perform an analysis of the band strengths.

### 2.10. Mitochondrial Morphology Observation

The mitochondrial morphology was observed as previously described [10]. Mitochondria in the CMECs were tagged with MitoTracker Deep Red (100 nM) at 37°C for 30 min. This was followed by the observation of the mitochondria employing confocal microscopy (Leica TCS SP5, Wetzlar, Germany) with a 60 × 1.3 NA oil immersion objective. A laser with a wavelength of 633 nm was employed to activate mitochondrial fluorescence, and the emissions were captured at a wavelength range of 558–617 nm. The program ImageJ V1.8.0 was utilized to measure and compute the length of mitochondria as well as their aspect ratios.

### 2.11. Measurement of ROS and Oxidative Stress

The ROS production was detected as previously described [10].CMECs were incubated with 10 *μ*M DCFH-DA at 37°C for 30 min. Using confocal microscopy (Leica TCS SP5, Wetzlar, Germany) with a 40x objective, DCFH-DA fluorescence was observed at an excitation wavelength of 488 nm and an emission wavelength ranging from 501 to 563 nm.

### 2.12. Autophagic Flux Assay

As per our earlier description, for determining the level of autophagy flux, Ad-mCherry-GFP-LC3B (Beyotime, Shanghai, CHINA) was used to transfect CMECs for 24 h [10]. Intense red fluorescent LC3 proteins revealed that autophagosomes became engulfed in the lysosomal acidic microenvironment to produce autolysosomes, which indicated a smooth autophagy flux. Intense yellow fluorescent LC3 proteins, on the other hand, indicated that autophagosomes were unable to be transformed into autolysosomes, which suggested that autophagy was inhibited.

### 2.13. Exosome Extraction

According to an earlier finding [18], the ultracentrifugation technique was employed to extract exosomes successfully. After centrifuging the cell specimens for 24 h at a speed of 10,000 × g and a temperature of 4° C, the supernatant was passed through a filter membrane with a pore size of 0.22 *μ*m. Then, the filtrate was centrifuged at 120000 × g for 2 h at 4°C. After that, the supernatant was collected with care, and the precipitate was rinsed with an equal volume of cold PBS before being centrifuged at a speed of 120000 × g for 2 h at 4°C. The sediment was reconstituted in 200 *μ*L of cold PBS and then placed in an ice bath at -80° C for viewing it utilizing transmission electron microscopy (TEM) and detecting proteins. The ZetaView SP2 program (Particle Metrix, Germany) was utilized to conduct an analysis of the exosomes' dimensions as well as their concentrations. To perform immunological blotting testing, identical quantities of exosome supernatant were placed into each well. The number of exosomes that were available was determined with the markers CD63 and TSG101.

### 2.14. TEM Imaging

To identify exosomes, 20 *μ*L of exosome suspension was placed on a fixed carbon mesh and let remain at room temperature for 20 min. After this period of time, the exosome suspension comprising the surplus discharge was carefully eliminated. After that, 20 *μ*L of phosphotungstic acid with a concentration of 2% was poured onto the carbon mesh, and it was allowed to rest for 20 s prior to transferring into a glass plate, which was covered with a filter membrane and maintained there until TEM inspection was carried out.

### 2.15. Statistical Analysis

All statistical calculations were carried out using R (version 3.6.3). Continuous variables were compared using Student's *t*-test for variables with normal distribution or the Mann–Whitney *U*-test for variables with an irregular distribution. In R, the “glmnet” tool was employed for the LASSO regression evaluation, whereas the “e1071” tool was employed for SVM technique assessment. Utilizing ROC curve modeling, the diagnostic accuracy of the included predictive biomarkers was determined. Spearman's correlation was utilized to investigate the connection between gene biomarker expression and immunological cell infiltration. Each statistical test was two-tailed, and *p* < 0.05 was utilized to determine statistical significance.

## 3. Results

### 3.1. Functional Correlation Analysis of the DEGs in AMI

Blood samples of CECs from 49 AMI patients and 50 healthy controls in the GEO dataset (GSE66360) were examined in this research. A sum of 122 DEGs were obtained: the expressions of 114 genes were significantly upregulated, and that of eight genes were reduced significantly (Figure 1).

To discover the roles of DEGs, enrichment studies of DO pathways were performed. The findings demonstrated that arteriosclerosis, arteriosclerotic cardiovascular illness, bacterial contagious sickness, coronary artery disorder, and myocardial infarction were strongly linked to DEG-enriched disorders (Figure 2(a)). GO studies revealed that the majority of the biological functions were associated with neutrophil stimulation in immunological reaction, cytokine generation, and leukocyte chemotaxis (Figure 2(b)). The IL-17 signaling pathway, lipid and atherosclerosis, tumor necrosis agent signaling pathway, and cytokine–cytokine receptor interactions dominated the enriched KEGG pathways (Figure 2(c)). These outcomes significantly imply that the immunological reaction is a crucial factor in AMI.

### 3.2. Identification and Verification of GABARAPL1 (GEC1) Gene as a Diagnostic Mitochondrial Biomarker for AMI

Two methods were utilized to identify possible biomarkers.

The LASSO regression approach was employed to filter down DEGs, resulting in the discovery of 17 factors as predictive biomarkers for AMI (Figure 3(a)). By using the SVM-RFE technique, a collection of 40 DEG characteristics was identified (Figure 3(b)). Between these two methods, nine overlapped characteristics (NR4A2, GABARAPL1, CLEC4D, ITLN1, SNORD89, ZFP36, CCR2, and EFEMP1) were identified (Figure 3(c)). We observed that GABARAPL1 (GEC1), an essential mitochondrial-related gene, may have a crucial part in AMI (Figure 3(d)). Using the GSE60993 and GSE123342 datasets, the GEC1 expression pattern in the peripheral circulation was validated to give more accurate outcomes. Investigation of the GSE60993 data revealed that the expression pattern of GEC1 was significantly greater in ST-segment elevation myocardial infarction (STEMI) than in non-STEMI, unstable angina (UA), and normal controls (Figure 3(e)). GSE123342 dataset analysis showed that GEC1, as a mitochondrial biomarker, was especially suitable for the acute attack of AMI than for stable coronary artery disease (CAD) and long-term post-MI (Figure 3(f)). Subsequently, GEC1 was utilized to construct predictive modeling employing a logistic regression technique in the metadata cohort, and the diagnostic capacity of GEC1 in differentiating AMI from control cases was found to have a satisfactory predictive value (AUG: 0.936, 95% CI: 0.882–0.977) (Figure 3(g)), suggesting that GEC1 may be a high-diagnostic feature mitochondrial biomarker for AMI.

### 3.3. High GEC1 in Blood CECs Is Due to Injured Cardiac CMECs Exfoliation Whose GEC1-Mediated Autophagy Is Overactivated after AMI

We further verified the expression of GEC1 in AMI rats. CECs were extracted from whole rat blood, and the expression of GEC1 in CECs was detected by flow cytometry. The data showed that the GEC1-positive expressed CECs in the blood of AMI group accounted for 93.47%, which was significantly higher than the 52.42% in the healthy group (*p* < 0.05) (Figure 4(a)). These outcomes were consistent with the bioinformatics analysis of the clinical data (Figure 1).

To explore the internal relationship between high expression of GEC1 in blood CECs and the occurrence of AMI, we detected the expression of GEC1 (labeled with FITC-GABARAPL1) in myocardial microvascular endothelial cells (CMECs, labeled with PE-CD31) in the heart tissue. The findings declared that the expression of GEC1 in cardiac CMECs was significantly elevated in AMI rats (*p* < 0.05) (Figure 4(b)). Immunofluorescence images further confirmed the high expression of GEC1 in the heart of AMI rats (Figure 4(c)). In addition, western blotting findings also declared that the LC3 II/I ratio was significantly upregulated in the hearts of AMI rats (Figure 4(d)), suggesting that GEC1-mediated autophagy might be overactivated in the heart of AMI.

### 3.4. The Oxidative-Damaged Mitochondria Block GEC1-Mediated Autophagy Flux and Are Released by Exosomes in Exfoliated Cardiac CMECs and Blood CECs

We constructed hypoxia-induced CMECs to simulate an AMI model at the cellular level. The confocal images showed that the mitochondrial length, as well as aspect ratio, was significantly decreased after hypoxia in CMECs (*p* < 0.05), and the ROS development in hypoxia-CMECs was also significantly increased (*p* < 0.05) (Figure 5(a)), indicating that hypoxia induced severe mitochondrial damage and oxidative stress in cardiac CMECs. In addition, autophagic flux detection showed that the number of autophagosomes significantly elevated (*p* < 0.05), but autolysosome number exhibited no increase correspondingly in CMECs that was hypoxia-induced (*p* > 0.05) (Figure 5(b)), implying that damaged lysosomes could not degrade many autophagosomes containing mitochondrial fragments in CMECs after hypoxia. However, autophagic flux was significantly improved after GEC1-shRNA treatment in hypoxia-CMECs (*p* < 0.05) (Figures 5(b)).

Interestingly, TEM results showed that blood CECs from AMI group released much more exosomes/microvesicles than that in the normal group (*p* < 0.05) (Figure 5(c)). Western blotting results declared that the expression of exosome biomarkers, such as TSG101 and CD63, was significantly increased in hypoxia-induced CMECs (*p* < 0.05), and the GEC1 expression was also increased in exosomes from hypoxia-induced CMECs (*p* < 0.05) (Figure 5(d)). The present findings declare that numerous undegraded autophagosomes containing damaged mitochondrial fragments in exfoliated cardiac CMECs and blood CECs could be released by exosomes in AMI.

### 3.5. The Exosome Burst Stimulates NLRP3 Inflammasome Production and Activates Vascular Inflammatory Response after AMI

To detect the effects of exosome/microvesicle burst in blood CECs after AMI, we explored the immune cell infiltration and found that the percentages of memory B cells (*p* = 0.047), CD4+ resting memory T cells (*p* < 0.001), gamma-delta T cells (*p* < 0.001), and excited natural killer (NK) cells (*p* < 0.001) significantly decreased after AMI, whereas the proportions of CD4^+^-activated memory T cells (*p* = 0.003), resting NK cells (*p* = 0.001), monocytes (*p* < 0.001), stimulated mast cells (*p* < 0.001), and neutrophils (*p* < 0.001) significantly increased after AMI (Figure 6(a)). We then performed a correlation analysis between GEC1 levels and immunological cell infiltration after AMI. The results showed that high GEC1 in blood CECs was strongly related to enhanced monocyte (*R* = 0.58, *p* < 0.001), activated mast cells (*R* = 0.41, *p* < 0.001), neutrophils (*R* = 0.40, *p* < 0.001), CD4^+^-activated memory T cells (*R* = 0.31, *p* = 0.002), and resting NK cells (*R* = 0.29, *p* = 0.004) and negatively correlated with the decreased proportion of CD4^+^ resting memory T cells (*R* = −0.56, *p* < 0.001), gamma-delta T cells (*R* = −0.48, *p* < 0.001), and stimulated NK cells (*R* = −0.37, *p* < 0.001) after AMI (Figures 6(b) and S1). These results suggest that high GEC1 in blood CECs may be tightly connected with the immune-inflammatory reaction in monocytes as well as neutrophils after AMI.

We further screened DEGs in AMI with immune-related gene clusters and inflammation-related gene clusters. The Venn diagram showed that 23 DEGs were related to the immune-inflammatory response in AMI (Figure 7(a)), including EDN1, CD14, PTAFR, LYN PLAUR, FPR1, C5AR1, AQP9, CSF3R, ICAM1, TLR2, CCRL2, NFKBIA, NAMPT, CXCL8, CCL20, NLRP3, IL1B, HBEGF, EREG, ADM, FFAR2, and LIF (Figure 7(b)). Notably, NLRP3, a hotspot inflammasome marker, was overactivated in the blood of AMI patients (Figure 7(c)). We further isolated immune monocytes, the proportion of which have been proven to be positively correlated with high GEC1, in AMI rats. The flow cytometry results showed that the NLRP3-positive monocytes in AMI group accounted for 93.18%, implying a significant rise contrasted with that of 54.41% in the healthy group (*p* < 0.05) (Figure 7(d)). Western blotting results showed that the expression of NLRP3 and corresponding inflammation indicators, such as caspase-1 and IL-1*β*, was significantly increased in blood CECs after AMI (*p* < 0.05) (Figure 7(e)). After tail vein injection with AAV2-shGEC1 to reduce GEC1 expression in cardiac CMECs, the vascular inflammatory response induced by NLRP3 inflammasomes could be markedly inhibited, suggesting the exosome burst with high GEC1 from blood CECs could stimulate NLRP3 inflammasome production and activates vascular inflammatory response after AMI.

## 4. Discussion

Acute myocardial ischemia (AMI) is the main reason of cardiovascular disease that leads to impairment and mortality all over the world every year [19]. Therefore, quick and correct identification of AMI is the essential stage for improving the prognosis of AMI patients [20]. Recently, with microarray technology and integrated bioinformatics investigation, many studies were conducted to discover unique genes or noncoding RNAs that can be used as diagnostic and prognostic biomarkers of AMI [21, 22]. However, these studies have primarily focused on inflammation and signaling cascade, and few have focused on the aberrantly expressed genes related to oxidative-damaged mitochondria and oxidative stress in AMI. Our study elucidated the process of vascular inflammation caused by myocardial ischemia from the perspective of mitochondrial quality imbalance and preliminarily explained the mechanism through the autophagic-exosome manner [23] in the cardiovascular system.

Mitochondria are essential organelles involved in several processes, such as maintaining cellular ion and energy balance, cell growth and death, etc. Mitochondrial quality imbalance and oxidative stress have been found in many tissues after acute ischemic/hypoxic injury [8]. Our previous study also demonstrated that the number of copies of mitochondrial DNA increased significantly in the superior mesenteric arteries (SMAs) after ischemia, and mitochondrial dynamics changed in primary vascular smooth muscle cells from rat SMAs after hypoxia [10]. In keloid fibroblasts under hypoxia, the mitochondrial complex activities significantly decreased, and the mitochondria were characterized by swelling, cristae effacement, and oxidative stress [24]. In Caco-2 cells, ischemia/reperfusion (I/R) induces severe mitochondrial oxidative damage and apoptosis [25]. In cardiomyocytes, the loss of regularity of mitochondrial striation and membrane integrity were found after I/R [26]. Due to mitochondrial quality imbalance being closely related to the establishment and prognosis of ischemic heart disorder, it is essential to determine possible predictive mitochondrial biomarkers for AMI and examine their roles in AMI.

To detect how markers in the blood can correlate with oxidative-damaged mitochondria in the heart, we selected circulating endothelial cells (CECs) as the target of our study. Meanwhile, cardiac microvascular endothelial cells (CMECs) are among the most abundant cells in the heart and actively participate in cardiac physiology and pathology [27, 28]. Under some pathological conditions, such as atherosclerosis, CMECs in the heart detach from the basement membrane, resulting in increased numbers of CECs within the blood, making CECs an ideal tissue to assess cell damage in the heart from blood [13, 29].

Using the public GEO dataset (GSE66360), 122 DEGs were detected with 114 elevated and eight decreased genes. DO pathway enrichment, GO, and KEGG pathway analyses significantly imply that the immunological reaction takes a key part in AMI, consistent with previous findings, which demonstrated that inflammation and immune responses are involved in AMI [30–32]. Further analysis according to two machine learning methods identified nine genes as potential diagnostic markers, of which GABARAPL1 (GEC1) was the only diagnostic mitochondrial biomarker for AMI. GABARAPL1 (GEC1), similar to GABARAP, engages with the GABAA receptor and tubulin as well as stimulates tubulin polymerization. Not only are the GABARAP group members (GABARAP, GABARAPL1, and GABARAPL2) and their similar homologs (LC3 and Atg8) engaged in the transportation of proteins or vesicles, but they are also involved in a wide range of mechanisms, including autophagy, apoptosis, cell growth, and tumorigenesis [33]. Nevertheless, in these given parallels, GABARAPL1 (GEC1) shows a control that is distinct from other GABARAP-related members. The study by An et al. [34] showed that GEC1 is essential for autophagosome maturation through the regulation of mitochondrial homeostasis. Boyer-Guittaut et al. [35] also demonstrated that GEC1 is essential for ensuring proper autophagic flux and performs an important function in controlling cell bioenergetics and metabolism, which was similar to our findings.

We found that mitochondria were seriously damaged and presented oxidative stress in hypoxia-induced CMECs, and GEC1 expression and the number of autophagosomes increased significantly, indicating that GEC1-mediated mitophagy was enhanced after hypoxia in CMECs. However, there was no increase in the number of autolysosomes. In contrary, we found that many more exosomes were released in exfoliated cardiac CMECs and blood CECs after AMI or hypoxia. Recently, studies have shown that, in addition to mitophagy, damaged mitochondria can also be packed into extracellular vesicles to be ejected from the cell. The study of Nicolas-Avila et al. [36] showed that dysfunctional mitochondria in cardiomyocytes could be ejected through a process driven by the cardiomyocyte's autophagy machinery and finally be eliminated by macrophages. The research of Crewe et al. [37] declared that adipocytes released secretory extracellular vesicles containing damaged mitochondria into circulation in response to energetic stress, which is taken up by cardiomyocytes and induces transient mitochondrial oxidative stress in cardiac tissue. The research of Souza et al. [37] declared that microvesicles transferred polarized mitochondria to the recipient's brain endothelial cells in culture and neurons in acute mouse brain cortical and hippocampal sections and elevated endothelial cell survivability under ischemic settings. The study of Ikeda et al. [38] showed that mitochondria-rich extracellular vesicles from autologous stem cell-derived cardiomyocytes restored the energetics of the ischemic myocardium. The study of Keulers et al. [39] showed that GEC1 is required for EV cargo loading and secretion. Based on these findings, we hypothesized and confirmed that the oxidative-damaged mitochondria block GEC1-mediated autophagy flux and are released by exosomes in exfoliated cardiac CMECs and blood CECs after AMI.

Inflammation plays an essential role in heart disease progression, and dysfunctional mitochondria are critical players in inflammation [40]. The study of Oka et al. [41] showed that mitochondrial DNA that escapes from autophagy cell-autonomously resulted in Toll-like receptor 9-mediated inflammatory reactions in cardiomyocytes. The study of Zhou et al. [42] showed that blockade of mitophagy caused the accumulation of oxidative-damaged mitochondria and activated the NLRP3 inflammasome, which was consistent with our results in this study. As per the correlation examination between GEC1 and infiltrating immunological cells after AMI, we found that high GEC1 in blood CECs might be closely associated with the immune-inflammatory response after AMI, suggesting that high GEC1 in exfoliated cardiac CMECs and blood CECs could activate vascular inflammatory responses by stimulating NLRP3 inflammasome production after AMI.

The limitations of this study are as follows: (1) In this paper, we only focus on the effects of GEC1-mediated mitochondrial damage and exosome burst in exfoliated cardiac CMECs on NLRP3 inflammasome and vascular inflammatory response after AMI, whether other cell types in heart tissues, such as macrophages and monocytes, participate in this regulation process need further investigation. (2) Due to ethical constraints, the experiments are only verified at the animal and cellular levels. In the next step, we will then collect clinical blood samples for further analysis and exploration.

## 5. Conclusion

In summary, oxidative-damaged mitochondria in cardiac CMECs activate GABARAPL1- (GEC1-) mediated autophagosomes but block autophagy flux after acute myocardial ischemia (AMI). The exfoliated cardiac CMECs evolve into abnormal blood CECs, and the undegraded GEC1 autophagosomes produce a large number of NLRP3 inflammasomes by exosome/microvesicle burst, stimulating the increase in monocytes and neutrophils and ultimately triggering vascular inflammation after AMI (Figure 8).

## Figures and Tables

**Figure 1:** DEGs between AMI and control samples. (a) Heatmaps of DEGs between AMI and control samples. (b) Volcanic map showing DEGs between AMI and control samples. Red dots exhibit significantly increased gene expression. Green dots exhibit significantly reduced gene expression. Block dots show non-DEGs.

**Figure 2:** Functional enrichment analyses of DEGs between AMI and control samples. Functional enrichment examinations of differentially expressed genes between AMI and control samples via (a) DO pathway enrichment analyses, (b) GO analyses, and (c) KEGG pathway enrichment analyses.

**Figure 3:** Screening process of diagnostic biomarker candidates for AMI diagnosis. Feature selection via (a) the LASSO regression algorithm and (b) SVM-RFE algorithm. (c) The Venn diagram shows nine potential diagnostic markers shared by the LASSO and SVM-RFE algorithms. (d) The Venn diagram demonstrates that GEC1 is the only mitochondria-related gene in the nine potential diagnostic markers. Validation of the expression of GEC1 in the (e) GSE60993 and (f) GSE123342 datasets. (g) The receiver operating characteristic (ROC) curve of GEC1.

**Figure 4:** The expression of GEC1 in the blood circulating endothelial cells (CECs) and heart cardiac microvascular endothelial cells (CMECs) after AMI. Flow cytometric analysis of the expression of GEC1 (a) in CECs and (b) in CMECs after AMI. (c) Immunofluorescence analysis of the expression of GEC1 in heart tissue after AMI (bar = 50 *μ*m). (d) The LC3 II/I ratio and the protein expression of GEC1 in the heart of AMI rats. (a) *p* < 0.05 compared with the normal group.

**Figure 5:** The detection of mitochondrial morphology, oxidative stress, autophagy flux, and exosome release in CMECs after AMI. (a) Mitochondrial morphology (bar = 25 *μ*m) and ROS production (bar = 50 *μ*m) in normal and hypoxia-CMECs. The length and aspect ratio of mitochondria were analyzed using the ImageJ software. The fluorescence intensity of DCFH-DA reflects the ROS production and oxidative stress. (b) Immunofluorescence images showing autophagy flux labeled by mCherry-GFP-LC3B in CMECs (bar = 10 *μ*m). (c) Transmission electron microscopic images show more exosomes being released after hypoxia treatment (bar = 100 nm). (d) Western blot analysis shows the effects of hypoxia on the expression of CD63, TSG101, and GEC1. (a) *p* < 0.05 compared with the normal group, (b) *p* < 0.05 compared with the hypoxia group.

**Figure 6:** The relationship between GEC1 expression in blood CECs and immune cell infiltration after AMI. (a) Comparison of 22 immune cell subtypes between AMI and normal tissues. Blue and red colors represent normal and AMI samples, respectively. (b) Correlation analysis between GEC1 and infiltrating immune cells after AMI.

**Figure 7:** The effects of GEC1 in blood CECs on NLRP3 inflammasome production after AMI. (a) Venn diagram showing 23 DEGs shared by immune-related gene cluster and inflammation-related gene cluster in AMI. (b) Heatmaps of the 23 DEGs related to immune and inflammation in AMI. (c) The expression of NLRP3 in blood after AMI is based on GSE66360 database. (d) Flow cytometric analysis of the expression of NLRP3 in blood monocytes after AMI. (e) Western blot analysis shows that the expression of NLRP3 and corresponding inflammatory factors were significantly increased in blood CECs after AMI, which was markedly inhibited by shGEC1. (a) *p* < 0.05 compared with the normal control group, (b) *p* < 0.05 compared with the AMI group.

**Figure 8:** Schematic diagram of oxidative-damaged mitochondria activating GEC1-induced NLRP3 inflammasomes in an autophagic-exosome manner after acute myocardial ischemia.

## Data Availability

The data that support the findings of this study are available from the corresponding authors upon reasonable request.

## Supplementary Materials

Supplementary Materials Figure S1 Correlation analysis between GEC1 expression and (A) monocytes, (B) activated mast cells, (C) neutrophils, (D) CD4 memory-activated T cells, (E) resting NK cells, (F) CD4 memory-resting T cells, (G) gamma delta T cells, and (H) NK cells activated after acute myocardial ischemia.
